The article "Indole-3-Carbinol Inhibits Nasopharyngeal Carcinoma Growth through Cell Cycle Arrest In Vivo and In Vitro" was retracted in 2022. Reasons: ethical violations by an author; a breach of policy by an author; concerns about the data.

# Indole-3-Carbinol Inhibits Nasopharyngeal Carcinoma Growth through Cell Cycle Arrest *In Vivo* and *In Vitro*

**DOI:** 10.1371/journal.pone.0082288

**Published:** 2013-12-16

**Authors:** Zhe Chen, Ze-Zhang Tao, Shi-Ming Chen, Chen Chen, Fen Li, Bo-kui Xiao

**Affiliations:** Department of Otolaryngology Head and Neck Surgery, Renmin Hospital of Wuhan University, Wuhan, China; Taipei Medical University, Taiwan

## Abstract

Nasopharyngeal carcinoma is a common malignant tumor in the head and neck. Because of frequent recurrence and distant metastasis which are the main causes of death, better treatment is needed. Indole-3-carbinol (I3C), a natural phytochemical found in the vegetables of the cruciferous family, shows anticancer effect through various signal pathways. I3C induces G1 arrest in NPC cell line with downregulation of cell cycle-related proteins, such as CDK4, CDK6, cyclin D1 and pRb. *In vivo*, nude mice receiving I3C protectively or therapeutically exhibited smaller tumors than control group after they were inoculated with nasopharyngeal carcinoma cells. The expression of CDK4, CDK6, cyclin D1 and pRb in preventive treatment group and drug treatment group both decreased compared with the control group. We conclude that I3C can inhibit the growth of NPC *in vitro* and *in vivo* by suppressing the expression of CDK and cyclin families. The drug was safe and had no toxic effects on normal tissues and organs.

## Introduction

Nasopharyngeal carcinoma (NPC), which is prevalent in Asia especially in the southern China, is a malignant tumor originating in the nasopharyngeal epithelium. It has close etiological association with the oncogenic Epstein–Barr virus (EBV), a strong etiological factor interacting with genetic predisposition and dietary intake of preserved foods. Radiotherapy (RT) is the mainstay treatment because of its high radiosensitivity, achieving a 5-year overall survival of 90% and 84% for early stage I and IIA disease, respectively.[1] Recurrence and distant metastasis remain the major causes of NPC-related death, despite the most aggressive treatment currently available such as concurrent chemoradiotherapy. With increasing local control from the primary treatment of NPC, the predominant mode of failure is unquestionably distant metastases.[2]

Recent dietary and epidemiological studies have shown the beneficial effects of intake of fruits and vegetables in lowering the incidence of cancers. Indole-3-carbinol (I3C), a natural phytochemical found in the vegetables of the cruciferous family, shows anticancer activity by inducing apoptosis[3], [4] and cell cycle arrest[5], [6], exhibiting antimetastatic properties[3], [7] and inhibiting angiogenesis gene products[8]. The anticancer activity of I3C is also reflected in a number of signal transduction pathways associated with the inhibition of cell growth. Previous studies have evaluated the inhibition effects of I3C on the prosurvival PI3K/Akt[3], [8], [9] and nuclear factor-κB[10] signal transduction pathways. I3C also down-regulates mitogen-activated protein kinases (MAPK) expression[11]. In this study we demonstrate the potential effects of I3C on induction of cell cycle arrest in NPC cells *in vitro*, and characterize the proteins involved *in vitro* and *in vivo*. Moreover we evaluate the preventive and therapeutic effects of I3C in nasopharyngeal carcinoma.

## Materials and Methods

### Reagents

The human NPC cell line, 5-8F, CNE2 and human normal bronchial epithelial cell line 16HBE were purchased from the Cancer Research Institute of Sun Yatsen University (Guangzhou, China) [12]–[14] and conserved in our laboratory and stored in liquid nitrogen. Fetal bovine serum (HyClone, USA), RPMI 1640 medium, 0.25% trypsin solution (Invitrogen, USA), cell counting kit-8 (Dongji, Japan), Cyclin D1, CDK4, CDK6, pRb, Rb antibody and GAPDH antibody (Cell Signaling Technology, USA) were purchased from companies mentioned above.

### Cell culture and grouping

Human nasopharyngeal carcinoma cell line 5-8F and CNE2 and human normal bronchial epithelial cell line 16HBE were cultured in RPMI 1640, supplemented with 10% fetal bovine serum and 20 µg/ml ampicilin and kanamycin. All the cells were maintained in an incubator with 5% CO_2_ at 37°C. Cells in logarithmic growth phase were used in the experiment. I3C diluted in DMSO with a final concentration of 0 µM, 100 µM, 200 µM, 300 µM, 400 µM was added in the 5-8F, CNE2 and 16HBE group, and control group using the same vehicle.

### Cell proliferation assay

5-8F, CNE2 and 16HBE cells were seeded in 96 well plates with 1×10^3^ cells per well for normal culture. I3C with a final concentration mentioned above were added in the experimental groups. The experiments in each group were done in duplicate for 3 times, and a blank control was also used. After 0 h, 24 h, 48 h and 72 h culture, 10 µl of CCK-8 was added into each well and incubated at 37°C for 1 hour, and the absorbance value was detected at 450 nm.

### Propidium Iodide single staining for detection of cell-cycle distribution

After treatment with different concentrations of I3C mentioned above for 48 h, 5-8F, CNE2 and 16HBE cells were harvested by trypsinization and the cells in each group were washed twice with cold phosphate-buffered saline. 70% ethanol was used for overnight fixation; after centrifugation, cells were resuspended in 500 ul PBS. Then 20 µl of 0.5% TritonX-100 and 1 mg/ml of RNase were added. After standing for 30 min at room temperature, 5 µl of 1 mg/ml propidium iodide(PI) solution was added and incubated for 30 min at room temperature. Flow cytometry analysis on a FACStar (Becton-Dickinson, Mountain View, California, USA) was then performed to determine the cell-cycle distribution. Approximately 10,000 cells were examined for each sample, and the data were analyzed with CELLQuest software (BD Biosciences, USA).

### Western blot

The 5-8F and CNE2 cells and tumor xenograft in nude mice were harvested and lysed in the buffer containing 1% Nonidet-P40, protease inhibitor ‘cocktail’ (Roche) and 2 mM dithiothreitol. Lysates were resolved by 12% SDS-PAGE, transferred to nitrocellulose membranes, and immunoblotted with primary antibodies against cyclin D1, CDK4, CDK6, pRb, Rb and GAPDH. After immunoblotting with secondary antibodies, proteins were detected with enhanced chemiluminescence (ECL) reagent.

### Animal feeding and grouping

Female BALB/C nude mice (4–6 weeks old) were purchased from Beijing HuaFukang Biological Technology Co. Ltd. (HFK Bioscience, Beijing, China) and underwent adaptive feeding one week prior to the experiment. Nude mice feed contained 0.5% I3C and the conventional nude mice feed were manufactured by Beijing HuaFukang Biological Technology Co. Ltd. Animal welfare and xenograft tumor inoculation were performed as previously described [15], [16]. The animals were divided into three groups (each consisting of eight nude mice), including the preventive treatment group (nude mice fed with feed containing 0.5% I3C for two weeks before the inoculation of nasopharyngeal carcinoma cells), the drug treatment group (feed containing 0.5% I3C when nasopharyngeal carcinoma cells were inoculated) and the control group (fed with regular feed and inoculated with nasopharyngeal carcinoma cells). The duration of the experiment was 8 weeks. The short and long diameter of xenograft tumors in Week 2, 4, 6, 8 after the inoculation of nasopharyngeal carcinoma cells were measured for volume calculation and statistical analysis. Tumor volume was estimated by the following equation: volume  = 1/2*L*W^2^, where L is length and W is width.[17] Eight weeks after inoculation, the animals were sacrificed and the xenograft tumors, the heart, liver and kidney were preserved for further evaluation. This study was approved by the Animal Ethics Committee of Renmin Hospital of Wuhan University.

### Hematoxylin and eosin staining

Specimens of the xenograft tumor, the heart, liver and kidney were fixed by formalin for 24 hours, dehydrated by 70%, 80%, 90% ethanol for 3 hours respectively, and then 100% ethanol I for 2 hours, 100% ethanol II for 2 hours and vitrified by xylene I and xylene II for 20 minutes. After immersing in paraffin I and II for 40 minutes, the specimens were embedded and sliced. Staining was performed as follows: hematoxylin staining for 15 minutes, hydrochloric acid alcohol solution for 35 seconds decoloring, eosin staining for 10 minutes and 90% ethanol for 40 seconds decoloring. Then neutral balsam was used for mounting and the section was observed and photographed under the microscope.

### Statistical analysis

All values were expressed as mean± SEM. Statistical analyses were carried out by one-way ANOVA using the SPSS statistical software (SPSS16.0 Inc., Chicago, IL, USA). Probability values *(P-value)* <0.05 were considered as statistically significant.

## Results

### I3C inhibited the growth of nasopharyngeal carcinoma cells

We used CCK-8 method to study whether I3C could effectively inhibit the proliferation of carcinoma cells. Treatment with I3C significantly inhibited the proliferation of 5-8F and CNE2 cells (Fig. 1A and 1B) in a dose- and time-dependent manner. Specially, in 5-8F and CNE2 cell line the inhibition efficiency both exceeded 60% when the final concentration of I3C reached 300 µM after 72 h treatment; and it reached to about 90% and 70% when the concentration was 400 µM. Additionally, in order to explore the effects of I3C on the proliferation and division of normal human tissues and cells, the same experiments were performed in human bronchial epithelial cells 16HBE (Fig. 1C). The results showed that 400 µM of I3C had much less inhibitory effect on 16HBE cell proliferation, compared with nasopharyngeal carcinoma cell line 5-8F and CNE2.

**Figure 1:** The viability of cells after I3C treatment. The viability of nasopharyngeal carcinoma cells 5-8F, CNE2 and human bronchial epithelial cells 16HBE were detected by CCK-8 assay. (A,B) The proliferation of 5-8F and CNE2 cells were inhibited by I3C in a dose- and time-dependent manner. (C)The proliferation of 16HBE cells were not inhibited by I3C.

### I3C induced cell-cycle arrest in nasopharyngeal carcinoma cells

To determine the effect of I3C on cell cycle, we evaluated the cell cycle distribution of 5-8F and CNE2 cells after 48 hours treatment of I3C with different concentrations using PI staining. The results showed that the cell cycle of nasopharyngeal carcinoma cells re-distributed after the treatment. With the increase of I3C concentration, proportion of G0/G1phase cells increased significantly, proportion of G2/M phase cells significantly reduced and proportion of S phase cells had no significant change. In 5-8F cells, G0/G1phase cells increased from 44.7% to 65.1%, G2/M phase cells decreased from 35.6% to 14.7%, S phase cells differed from 19.8% to 20.3%. In CNE-2 cells, G0/G1phase cells increased from 39.2% to 54.3%, G2/M phase cells decreased from 33.9% to 18.1%, S phase cells differed from 26.7% to 27.4%. (Fig. 2A and 2B). However, when the concentration of I3C changed from 0 to 400 µM, each phase cells in 16HBE cell line did not elevate significantly (Fig. 2C).

**Figure 2:** The result of cell cycle distribution. The cell cycle distribution was detected by flowcytometry. (A,B)The proportion of G0/G1 phase cells increased and G2/M phase cells decreased in 5-8F and CNE2 cell lines as I3C concentration increased. (C)The proportion of all phase cells barely elevated in 16HBE cell line as I3C concentration increased. The data are presented as the mean± SEM. *p<0.05, compared to the proportion of each phase cells in 0 µM I3C treatment.

### I3C changed the expression of cell cycle related proteins after treatment in vivo and in vitro

The results shown above implicate that I3C had a significant regulatory role in the cell cycle of nasopharyngeal carcinoma cell lines. Therefore, we evaluated the expression of several key proteins involved in cell cycle regulation of nasopharyngeal carcinoma cells. It was observed that as I3C concentration increased, the protein expression levels of cyclin D1, CDK4, CDK6 and pRb were down-regulated in 5-8F and CNE2 cells (Fig. 3). Additionally, the expression of these proteins in the nude mice xenograft tumors of 5-8F and CNE2 from I3C preventive and I3C treatment groups decreased, as compared to the control group. (Fig. 4)

**Figure 3:** The expression of cell cycle related proteins in vitro. Key proteins related to cycle regulation were detected by WB. As I3C concentration increased, cyclin D1, CDK4, CDK6 and pRb protein expression in 5-8F(A) and CNE2(B) cell line were down-regulated. The data are presented as the mean± SEM.

**Figure 4:** The expression of cell cycle related proteins in vivo. Cyclin D1, CDK4, CDK6 and pRb protein expression were down-regulated in the xenograft tumors of 5-8F(A) and CNE2(B) in I3C preventive and I3C treatment groups compared to the control group. The data are presented as the mean± SEM.

### I3C changed the expression of MAPK and NF-κB signaling after treatment in vivo and in vitro

The expression of MAPK proteins and NF-κB were detected in cells and xenograft tumors. P-ERK1/2, P-JNK, P-P38 and NF-κB(p65) were down-regulated in 5-8F and CNE2 cells when the concentration of I3C increased (Fig. 5). The expression of these proteins in the nude mice xenograft tumors of 5-8F and CNE2 from I3C preventive and I3C treatment groups also decreased, as compared to the control group. (Fig. 6)

**Figure 5:** The expression of MAPK and NF-κB proteins in vitro. The expression of MAPK and NF-κB signaling decreased *as* I3C concentration increased in 5-8F(A) and CNE2(B). The data are presented as the mean± SEM.

**Figure 6:** The expression of MAPK and NF-κB proteins in vivo. MAPK and NF-κB proteins expression were down-regulated in the xenograft tumors of 5-8F(A) and CNE2(B) in I3C preventive and I3C treatment groups compared to the control group. The data are presented as the mean± SEM.

### Anti-tumor efficacy of I3C in nude mice

The anti-tumor effects of I3C were studied by *in vivo* animal experiments. The tumor volumes increased rapidly in the control group, which was given only conventional nude mice feed. In the 8th week of the experiment, the mean volume of the xenograft tumor in the nude mice of the 5-8F/CNE2 cell control group, I3C drug treatment group and I3C preventive treatment group were(2266±543.46)/(2649±499.15) mm^3^, (1347±232.73)/(1478±257.09) mm^3^ and (623.1±201.76)/(717±232.03) mm^3^, respectively (Fig. 7).

**Figure 7:** Anti-tumor efficacy of I3C in nude mice. The effect of I3C on tumor growth of 5-8F(A) and CNE2(B) in xenograft nude mice. The data are presented as the mean± SEM. *p<0.05, compared to control group.

### Safety of I3C as an anti-tumor agent

To evaluate if I3C causes pathological damages to vital organs of the experimental animals during treatments, routine HE staining of the sections of the heart, liver and kidney of the nude mice in different groups was performed. No degeneration, necrosis or structural disorders in the heart, liver and kidney was observed in all groups, suggesting that the feed containing 0.5% I3C had no toxic or side effects on the heart, liver and kidney of the experimental animals (Fig. 8).

**Figure 8:** The result of HE staining of main organs of nude mice after I3C treatment. (A) HE staining of heart, (B) HE staining of liver, (C) HE staining of kidney.

## Discussion

It has been reported that the median survival time for an NPC patient with metastatic or advanced disease was only 5 to 11 months[18]. Although NPC is a radiosensitive tumor compared with other head or neck cancers, the high incidence of recurrence, lymph node spread and distant metastases cause poor prognosis[19]. Chemotherapy plays an important role in the treatment of NPC. The major problem of current chemotherapy is the high toxicity of the drugs being used[20]. Therefore, NPC chemotherapy needs drugs with improved efficacy and safety.

I3C is an active ingredient extracted from natural cruciferous plants. It shows significant anti-tumor effect in various tumor cells. It effectively induces cell cycle arrest in prostate[5], colon[9], breast[21] and lung[22] cancer cells. The studies of I3C in nasopharyngeal carcinoma were not sufficient. Zhu and Xu showed the effect of I3C in apoptosis in nasopharyngeal carcinoma *in vitro* and *in vivo* [23], [24]. In our study, I3C can inhibit the proliferation of human nasopharyngeal carcinoma cell lines 5-8F and CNE2, but not the human normal bronchial epithelial cell line 16HBE in our study. This phenomenon demonstrated that I3C suppressed the growth of tumor cells while exerting little effect on normal cells *in vitro*. We considered that I3C could inhibit the proliferation of carcinoma cells specially and it might be safe to normal cells. Thus, I3C used as an anti-tumor drug is promising.

On the basis of previous studies[25]–[27], our results demonstrated that I3C induced G0/G1 cell cycle arrest in the 5-8F and CNE2 cell line and this arrest was accompanied by the down-regulation of cyclin D1, CDK4, CDK6 and pRb in 5-8F and CNE2 cells *in vitro* and *in vivo*. The mechanism of cell cycle regulation is the reciprocity of cyclins, CDKs, and CDKIs[28]. CDKs are the core effectors in cell cycle progression. CDK activity is regulated through the association with their cyclin partners and CDKIs as well as by activating and inhibiting the phosphorylation events. CDK4/6 is associated with cyclin D and it phosphorylate Rb protein. They initiate progression at the restriction point in G1 phase[29]. Cyclin D/CDK4/6 activity occurs in mid-late G1 phase, and it is required for the hyperphosphorylation of the retinoblastoma gene product (pRb). The protein Rb controls progression at the late G1 restriction point and is a major regulator of the G1/S transition[30]. Alterations of any component of this pathway, such as overexpression of cyclin D related CDKs, or mutations to CDKs that affect p16 binding, will lead to Rb phosphorylation and subsequent progression from G1 to S phase[31], [32]. These alterations have been found in many human tumors, suggesting that inactivation of the cell cycle pathway may play an important role in their pathogenesis. The loss of p16 and p21 and the increase of CDK4 and cyclin D1 expression were observed in the NPC specimens compared with histologically normal nasopharyngeal epithelial (NPE), dysplastic NPE, and the matched adjacent epithelia of NPC[33].

MAPK signaling is mediated by ERK1/2, JNK and p38 MAPK, which are important in the control of cell proliferation, differentiation and transformation. NF-κB, a transcriptional factor, is critically involved in tumor progression due to its transcriptional regulation[34]. Moreover, NF-κB signaling pathway has been shown to block apoptosis which induced by death receptors and promote proliferation of cancer cells. Constitutive activation of NF-κB has been detected in various tumor cells [35]. These results suggested that the cell cycle arrest observed may be regulated through a MAPK pathway by transcriptional down-regulation of cell cycle proteins. Western blotting confirmed that I3C expression down-regulated several components of the MAP kinase and NF-κB pathway and in NPC cells and xenograft tumors. It also inhibits NPC cell growth and cell cycle progression from G1 to S phase in vitro, and suppresses NPC cell tumor formation in vivo. The most likely mechanism underlying the I3C-induced growth arrest involves down-regulation of MAP kinases and NF-κB pathway, which leads to reduction in G1-related CDKs, such as CDK4 and p-RB, and a decrease in cyclin D1 and CDK4 expression. [35].

In the current study normal diet containing 0.5% I3C was given in the preventive and treatment group. Eight weeks after the inoculation of tumor cells, the tumor volume was the smallest in I3C preventive treatment group, moderate in treatment group and the biggest in control group. Studies showed that I3C is unstable in acidic milieu such as gastric juice, thereby converting into several condensation products [36]. I3C exhibits biological activities such as anti-proliferative and pro-apoptotic against tumor or endothelial cells, but the effective concentrations of I3C used in those experiments were relatively high in vitro(>100 µM in most cases) [8], [37]–[40]. A previous study [41] detected I3C in tissues following the dosing of mice with 250 mg/kg I3C using an HPLC method. The maximum level of 28 µM I3C was observed at 15 min. Pharmacokinetic studies in mice and humans demonstrated that the concentration of I3C in plasma fell below the limit of detection within 1 h [42], [43]. The average amount of I3C in the mice in preventive and treatment group intake was close to 250 mg/kg. It indicated that the concentration of I3C in plasma was approximate 28 µM. In concentrations much less than 300 µM, I3C could inhibit the growth of xenograft tumor in those two groups. It means that I3C could inhibit the growth of tumor effectively in vivo. The possibility is that in vivo metabolites, are more active than I3C against nasopharyngeal carcinoma cells. Clinical studies have established that ingestion of 400 mg of I3C twice daily is well tolerated [44] http://www.sciencedirect.com/science/article/pii/S095528631200068X - bb0165. In the present study, mice were treated with I3C orally at a dosage of about 250 mg/kg per day, which is equivalent to a dose of 20.3 mg/kg in an average adult human[45]. This dose is within the range that has been used in clinical trials. Moreover, since the amount of inoculated nasopharyngeal carcinoma cells in this experiment was large (approximately 2×10^6^), it was unlikely to be completely prevented by I3C. The initial number of tumor cells due to mutation in the human body was small and stable blood plasma concentrations of I3C could destroy the majority of mutated tumor cells, which might play an important role in the prevention of nasopharyngeal carcinoma tumor.

In summary, our study showed that I3C effectively inhibited nasopharyngeal carcinoma cell growth. As a natural ingredient, I3C caused little damage to normal cells and tissues, and was relatively safe to use. The results of animal experiments suggested that I3C had certain tumor preventive effect and inhibited the formation and development of tumors. In the future, we will focus on the therapeutic effect of I3C in recurrent nasopharyngeal carcinoma.
